# A Network with Composite Loss and Parameter-free Chunking Fusion Block for Super-Resolution MR Image

**DOI:** 10.1155/2023/4959130

**Published:** 2023-06-12

**Authors:** Qi Han, Mingyang Hou, Hongyi Wang, Zicheng Qiu, Yuan Tian, Sheng Tian, Chen Wu, Baoping Zhou

**Affiliations:** ^1^School of Intelligent Technology and Engineering, Chongqing University of Science and Technology, Chongqing 401331, China; ^2^College of Information Engineering, Tarim University, Alar 843300, China

## Abstract

MRI is often influenced by many factors, and single image super-resolution (SISR) based on a neural network is an effective and cost-effective alternative technique for the high-resolution restoration of low-resolution images. However, deep neural networks can easily lead to overfitting and make the test results worse. The network with a shallow training network is difficult to fit quickly and cannot completely learn training samples. To solve the above problems, a new end-to-end super-resolution (SR) method is proposed for magnetic resonance (MR) images. Firstly, in order to better fuse features, a parameter-free chunking fusion block (PCFB) is proposed, which can divide the feature map into *n* branches by splitting channels to obtain parameter-free attention. Secondly, the proposed training strategy including perceptual loss, gradient loss, and *L*1 loss has significantly improved the accuracy of model fitting and prediction. Finally, the proposed model and training strategy take the super-resolution IXISR dataset (PD, *T*1, and *T*2) as an example to compare with the existing excellent methods and obtain advanced performance. A large number of experiments have proved that the proposed method performs better than the advanced methods in highly reliable measurement.

## 1. Introduction

MRI is a noninvasive imaging technology in vivo that uses the phenomenon of magnetic resonance to obtain molecular structure and thus information about the internal structure of the human body. MRI not only provides more information than many other imaging techniques in medical imaging, but it can also directly make cross-sectional, sagittal, coronal, and various oblique images of the body, which does not produce the artifacts in CT detection, does not require contrast injection, does not have ionizing radiation, and has less adverse effects on the body. MRI is very effective in detecting intracerebral hematomas, extracerebral hematomas, brain tumors, and other diseases. Of course, MRI has its shortcomings [1]. It is relatively slow, has less spatial resolution than CT, has motion artifacts, etc. Therefore, obtaining high-resolution MRI images has become the direction of current research.

High-resolution MRI can not only clearly show the relationship between tumor and surrounding tissues but also the anatomical structure of the brain. It has high application value in the early and middle stages of diagnosis [2].

However, the generation of high-resolution MRI images is odnften influenced by many factors, such as hardware equipment, imaging time, the motion of the human body, and the effect of environmental noise. Therefore, in order to perform effective high-resolution restoration of the low-resolution images obtained by MRI, image super-resolution is an effective and cost-effective excellent technique to improve the spatial resolution of MR images. This technique offers the feasibility of a high signal-to-noise ratio and high-resolution reconstruction of low-resolution MRI images [3].

The traditional SR algorithms include interpolation-based and reconstruction-based methods, which are generally difficult to reconstruct from the high-frequency detailed information of the image, more complicated to compute, and take longer time to reconstruct [4]. In order to solve these problems, scholars have applied deep learning to SR reconstruction in recent years and made a lot of breakthroughs, and nowadays, SR algorithms based on deep learning have occupied the mainstream position of SR algorithm research. In the field of medical images, deep learning-based SR algorithms can obtain prior knowledge from medical image training set data and reconstruct low-resolution images into high-resolution images using neural networks based on this information.

In recent years, with the continuous development of deep learning [5–8], many advanced deep learning-based SR methods have emerged in the field of SR image [9, 10], enabling the performance and efficiency of SR image to be continuously enhanced. Super-resolution convolutional neural network [11] and fast super-resolution evolutionary neural network [12] were pioneering works of deep learning in the field of super-resolution reconstruction. They use a convolutional neural network (CNN) for super-resolution image reconstruction for the first time. Subsequently, on the basis of this pioneering work, researchers proposed many new super-resolution image networks to further improve the model performance, such as deeply recursive convolutional network [13] and deep recursive residual network [14] based on recurrent neural networks and super-resolution using very deep convolutional networks [15]. FFTI [16] was a fine inpainting method which is an incomplete image inpainting method based on feature fusion and two-step inpainting. However, most of these methods were aimed at natural images and are not suitable for medical images.

Recently, many literature studies in the field of medical images have also proposed many SR methods for medical images, such as [17–21]. However, unlike ordinary images, high-quality medical image datasets are relatively scarce, and most of the images are gray-scale images, and the images are relatively single. Using this data set to train a model with a deep network layer will easily lead to overfitting and make the test result worse. A model with a shallow training network will be difficult to fit quickly and cannot learn the training samples completely. Therefore, SR medical images trained by a traditional network cannot meet the requirements of SR tasks.

Considering the above problems, in order to make a SR image model more suitable for medical image tasks, in this paper, we introduce residual learning and a parameter-free chunking fusion method to improve the above difficulties. In the stage of feature extraction, residual learning is designed similar to the residual network [22] to acquire features, which uses layerNorm [23] in the transformer for reference. LayerNorm is also used in residual learning to make the training smoother and avoid the impact of variance differences between different batches. Subsequently, a parameter-free chunking fusion block is used to better fuse features and perform effective feature enhancement. In the module, the feature graph chunking is divided into *n* branches for different information transmission, and then the SimAM [24] is performed on each branch to enhance the features of different branches, and finally the semantic information of different branches is integrated. SimAM can effectively enhance the feature on different branches and effectively integrate at the end. Moreover, SimAM has no parameters to learn and can improve the model performance without parameter training. In addition, in order to further accelerate model fitting and improve prediction accuracy, this paper proposes a composite loss to optimize the training strategy by combining perceptual loss, gradient loss, and *L*1 loss.

In order to solve the above problems, we have proposed corresponding solutions, to which the follow-up work mainly makes three contributions:

1. A parameter-free chunking fusion block (PCFB) model is proposed, which divides the feature map into *n* branches for parameter-free attention and then integrates the feature information of different branches, so as to better fuse features and perform effective feature enhancement, which can improve the expression ability of the feature map without adding parameters, thereby improving the accuracy.
2. A composite loss for our SR method is proposed which combines perceptual loss, gradient loss, and *L*1 loss. The loss can further make the model pay attention to the impact of loss in different dimensions, thus enhancing the model's expressiveness.
3. A new end-to-end SR method for MR images is proposed, where the methods contain PCFB and composite loss, which can improve SR method performance more effectively and avoid overfitting.

The rest of this paper is organized as follows: Section 2 introduces some related work in this paper. The proposed methods and experimental results are described in detail in Sections 3 and 4, respectively. We conclude our thesis in Section 5.

## 2. Related Work

### 2.1. Super-Resolution in Deep Learning

With the development of deep convolutional neural networks (DCNN), research on super-resolution has made progress recently. For deep learning methods with SISR, fast response and reconstruction quality are important references for measuring super-resolution methods. Super-resolution convolutional neural network (SRCNN) [11] and fast super-resolution evolutionary neural network (FSRCNN) [12] were pioneering works of deep learning in the field of super-resolution reconstruction. The two neural networks first used bicubic interpolation to reduce and enlarge low-resolution images to obtain comparable super-resolution images. Then convolutional neural network was first introduced to achieve image reconstruction. In addition, the traditional SR method based on sparse coding can also be regarded as a deep convolutional network from the two networks, and compared with the traditional method, all sublayers in the two networks were optimized to give full play to the performance of each component. DRCN has a very deep recursion layer (up to 16 recursions), and recursive supervision and skip connections were further proposed by taking into account gradient disappearance/explosion. For deep models, the residual structure exhibits excellent performance. Therefore, the residual structure is introduced into the super-resolution method to make up for the shortcomings caused by gradient disappearance and gradient explosion. The deep super-resolution network (EDSR) [25] was inspired by the residual structure. Compared with the traditional residual structure, the residual blocks of EDSR discard unnecessary modules, thus constructing a multiscale depth super-resolution system (MDSR), which can reconstruct high-resolution images with different magnification factors in a single model. In addition, the SR robustness of images in complex scenes should also be focused on. A heterogeneous group SR CNN [9] contains multiple heterogeneous group blocks. These blocks increase the internal and external relations of different channels in a parallel way to cope with SR in complex scenarios. An enhanced super-resolution group CNN (ESRGCNN) [26] can fully fuse the correlation between wide channel features and retain the long-distance context dependence in the upsampling operation to obtain more accurate low-frequency information. Further, in order to solve the common problems in image super-resolution algorithms, such as image edge blurring caused by redundant network structure, inflexible selection of convolution kernel size, and slow convergence speed of training process, MFFN [27] used a lightweight fusion multilevel single image super-resolution method to achieve SISR.

### 2.2. Super-Resolution in Medical Imaging

The problem of super-resolution has been widely discussed in medical imaging. Due to limitations such as image acquisition time, low radiation dose, or hardware limitations, the spatial resolution of medical images is insufficient [28]. To solve this problem, Zhu et al. [29] proposed a method for arbitrary scale super-resolution (MIASSR) of medical images, where the method also combined meta-learning with GAN, which can be used for super-resolution at any magnification.

To get as many useful image details as possible, Bing et al. [20] proposed a SR method in medical imaging based on an improved generative adversarial network. This method can not only avoid the interference of high-frequency false information but also integrate the low-level feature constraints to train the model. Zhang et al. [21] proposed a fast medical image super-resolution method, in which subpixel convolution layer addition and mini-network replacement in the hidden layer were crucial to improving the speed of image reconstruction. Inspired by the super-resolution convolutional neural network method based on three hidden layers, Deeba et al. [18] proposed a wavelet-based microgrid network super-resolution method for medical images, where image restoration was speeded up by adding a subpixel layer to replace the small grid network on the hidden layer.

### 2.3. Attention Mechanism for Vision Tasks

Attention has arguably become one of the most important concepts in the field of deep learning. It was inspired by human biological systems, which tend to focus on unique parts when processing large amounts of information [30]. Liu et al. [31] proposed a multiattention domain module to weigh and reorganize the features; the channel and spatial domain information in the super-resolution method are effectively fused, and the quality of the super-resolution image is effectively improved. Wang et al. [32] proposed two new attention mechanisms: context-weighted channel attention and persistent spatial attention. The proposed attention modulates rich features by suppressing useless features and enhancing features of interest in a channel and spatial manner. Liu and Chen [33] made the following improvements on the basis of the super-resolution universal reverse network (SRGAN). Firstly, they added the channel attention (CA) module to the SRGAN network and increased network depth to better express high-frequency features. Secondly, the old batch normalization layer is deleted to improve network performance. Finally, the loss function is modified to reduce the influence of noise on the image.

## 3. Methods

### 3.1. Overview

In the image super-resolution task, our goal is to take the low-resolution (LR) image *I*_*LR*_ ∈ *ℝ*^*H*×*W*×*C*^ as the input of the super-resolution model and generate the super-resolution (SR) image *I*_*SR*_ ∈ *ℝ*^*H*×*W*×*C*^. While the general low-resolution image *I*_*LR*_ is obtained by downsampling the ground-truth of the high-resolution image *I*_*HR*_ ∈ *ℝ*^*H*×*W*×*C*^. We expressed the super-resolution model as *G* and the parameter as *θ*_*G*_. The super-resolution task can be expressed as the following formula:

(1) $$\begin{array}{c} I^{SR}=G\left(I^{LR};\theta_{G}\right)\text{.} \end{array}$$

In order to make *I*_*SR*_ as similar to *I*_*HR*_ as possible, it is necessary to optimize the model *G* with the loss function *L*, and finally the optimal parameter *θ*_*G*_^*∗*^ is obtained. The objective formula is as follows:

(2) $$\begin{array}{c} \theta_{G}^{*}=\underset{\theta_{G}}{\mathrm{argmin}}E_{I^{SR}}L\left(I^{SR}-I^{HR}\right)\text{.} \end{array}$$

The proposed architecture of super-resolution is shown in Figure 1. Then, the details are given about the feature extraction block, parameter-free chunking fusion block (PCFB), and image reconstruction block. Finally, the composite loss and the training strategy are introduced to enhance the model's expressiveness.

### 3.2. Network Architecture

#### 3.2.1. Feature Extraction

The feature extraction part is composed of convolution, activation function, and residual block.

First, if the normal ReLU activation function is used, when the feature *x* is less than 0, *x* will be suppressed to 0, and the feature information will be lost. Therefore, we use PReLU [34] (parametric rectified linear unit) to replace ReLU. PReLU adds a learnable parameter on the basis of ReLU, which can adjust the activation function according to different experimental conditions. The formula is as follows:

(3) $$\begin{array}{c} PReLU\left(x_{i}\right)=\left\{\begin{array}{ll} x_{i}\text{,} & if\;x_{i}>0\text{;}\\ a_{i}x_{i}\text{,} & if\;x_{i}\leq 0\text{.} \end{array}\right. \end{array}$$

where *x* represents the the feature map, *a*_*i*_ ∈ [0,1] is a learnable parameter.

Second, if batch normalization (BN) is used, due to the difference in the mean and variance of data in the mini-batch, unstable statistical data may be brought [35], and instance normalization [36] can avoid the above small batch problems. However, the work reported in [37] shows that adding instance normalization does not always bring performance improvement, and manual adjustment is required. Therefore, we introduce layer normalization (LN), which was used by relevant papers of transformer [23] in the early stages. Many recent SOTA methods [38–40] also use this normalization. LayerNorm is independent of the batch size, so it will not be affected by the above problems, and there are no parameters that need to be manually adjusted in the instance normalization. Therefore, LN is introduced to stabilize the training and improve the performance. The normalization formula is as follows:

(4) $$\begin{array}{c} y=\frac{x-E\left[x\right]}{\sqrt{Var\left[x\right]+\epsilon }}*\gamma +\beta \text{,} \end{array}$$

where *x* represents the feature map, *ϵ* is a small constant, *𝔼*[*x*] is mean, Var[*x*] is variance, and *γ* and *β* is scale and shift. The same normalization method is used as BN, but the difference is that LN normalizes each single batch rather than normalizing all batches together like BN.

#### 3.2.2. Parameter-Free Chunking Fusion Block (PCFB)

In order to improve the propagation of feature information, Zhao et al. [41] designed module CSB to help the neural networks deal with hierarchical features with different attributes. Because CBF contains a large number of parameters that need to be learned and the fitting speed is slow, we propose PCFB that does not need to learn a large number of parameters on the basis of maintaining image quality. In PCFB, chunking and fusing are represented as channel splitting and channel merging, respectively.

The difference from CSB is that the size of the chunking is determined by the parameter *n*, where each input feature *x* is divided into *n* chunks, and each chunk *x*^*i*^ is the size of *H* × *W* × (*c*/*v*). Subsequently, in order to carry out targeted feature enhancement for each block of data, SimAM is used to process features of different blocks, and SimAM does not need redundant parameters to be learned, so the number of model parameters will not be increased.

*(1) Chunking and Fusing*. The input feature *x* can be divided into *n* chunks along the channel direction, and the dimension of each chunk is *H* × *W* × (*c*/*v*). It can be formally expressed as follows:

(5) $$\begin{array}{c} S\left(x\right)=x^{1},x^{2}\ldots x^{n},i=1,2,\ldots ,n\text{,} \end{array}$$

(6) $$\begin{array}{c} x=M\left(x^{1},x^{2}\ldots x^{n}\right),i=1,2,\ldots ,n\text{,} \end{array}$$

where *S*(·) is the chunking function which split feature map *x* into *n* chunks *x*_1_, *x*_2_ … *x*_*n*_. In contrast, *M*(·) is the fusing function, which can merge *x*_1_, *x*_2_ … *x*_*n*_ back to the original dimension use concat function.

*(2) Parameter-Free Attention*. Normally, spatial attention is often used for spatial information, while channel attention is often used for channel information to focus on feature information. However, in human eyes, spatial attention and channel attention coexist and jointly promote information selection in visual processing. Therefore, we need a three-dimensional attention to focus on the features in each channel and spatial position, so a parametric 3D attention SimAM is used to enhance the features of different chunks in the paper. The structure of the proposed method is shown in Figure 2.

SimAM evaluates the importance of each neuron by constructing an energy function *e*_*t*_^*∗*^. The lower the energy, the greater the difference between the neuron and surrounding neurons, and the higher the importance of features. The energy function is as follows:

(7) $$\begin{array}{c} e_{t}^{*}=\frac{4\left(\hat{\sigma^{2}}+\lambda \right)}{{\left(t-\hat{u}\right)}^{2}+2{\hat{\sigma }}^{2}+2\lambda }\text{,} \end{array}$$

where *t* is a neuron which means a pixel of feature map *x*, $\hat{u}$, and $\hat{\sigma }$ represent the mean and standard deviation of the characteristic map, respectively, and *λ* is a hyper parameter.

Therefore, the importance of neurons can be obtained by *e*_*t*_^*∗*^. In addition, the attention mechanism can be realized by weighting the feature map through the sigmoid function. The formula is as follows:

(8) $$\begin{array}{c} T\left(x\right)=sigmoid\left(\frac{1}{E}\right)⊗x\text{,} \end{array}$$

where ⊗ means element-wise multiplication, and *E* is the energy matrix containing all *e*_*t*_^*∗*^. This module does not introduce any additional training parameters, so it does not increase the original network parameters on the premise of improving performance.

*(3) Parameter-Free Chunking Fusion Block*. In order to better learn and enhance the features, we use equation (5) to obtain *n* chunks and then let each chunk pass through equation (8) alone for 3D weighted attention. Equation (6) is used to fuse them into the original size like equation (9). The process is shown in Figure 1.

(9) $$\begin{array}{c} x=M\left(T\left(x_{1}\right),T\left(x_{2}\right)\ldots T\left(x_{n}\right)\right),i=1,2,\ldots ,n\text{.} \end{array}$$

#### 3.2.3. Image Reconstruction Block

In order to change the image to the super-resolution size, the upsampling operation is required, and we build the image reconstruction part to realize it. As shown in Figure 1, image reconstruction includes 3 × 3 convolution, 1 × 1 convolution, PReLU, and PixelShuffle [42] layers.

The main function of PixelShuffle is to obtain high-resolution feature maps by multichannel recombination of low-resolution feature maps. As shown in Figure 3, the feature mapping of the *r*^2^ channels is recombined into the supersampling result of (*H∗r*) × (*W∗r*) of a single channel. Pixel shuffle transforms the feature map from low-resolution space to high-resolution space.

### 3.3. Our Composite Loss for Super-Resolution

#### 3.3.1. Conventional Loss

Most super-resolution methods use pixel loss to optimize the network. Pixel loss measures the pixel-wise difference between SR image and HR image, which contains *L*1 loss and *L*2 loss. Compared with *L*1 loss, *L*2 loss penalizes large errors but has a higher tolerance for small errors. In actual training, *L*1 loss [25, 43] shows better convergence than *L*2 loss. Finally, a higher peak signal-to-noise ratio (PSNR) index will be obtained, so it is the most widely used loss function in the super-resolution field. The formula is as follows:

(10) $$\begin{array}{c} L_{SR}^{L1}=E_{I^{SR}}{\left\|G\left(I^{LR}\right)-I^{HR}\right\|}_{1}\text{,}\\ L_{SR}^{L2}=E_{I^{SR}}{\left\|G\left(I^{LR}\right)-I^{HR}\right\|}_{2}\text{.} \end{array}$$

However, since such pixel loss does not consider the image quality, such as edges, textures, and high-frequency details, which may be too smooth to maintain sharp edges to obtain visual effects.

#### 3.3.2. Perceptual Loss

In order to incorporate high-level feature loss on the basis of pixel loss, perceptual loss [44] is introduced. The perceptual loss uses the pretrained VGG [45] network to extract the high-level features of the image and constructs the perceptual loss through the Euclidean distance between the HR image features and the SR image features to restore the perceptual quality of the image. The formula of perceptual loss is as follows:

(11) $$\begin{array}{c} L_{SR}^{Per}=E_{I^{SR}}{\left\|\phi_{i}\left(G\left(I^{LR}\right)\right)-\phi_{i}\left(I^{HR}\right)\right\|}_{1}\text{,} \end{array}$$

where *ϕ*_*i*_(·) denotes the *i*-th layer output of the VGG model.

#### 3.3.3. Edge-Aware Loss

In order to combine the loss of image edge information on the basis of pixel loss, we further introduce edge-aware loss [46]. In edge-aware loss, edges of the SR image and HR image are extracted according to the edge extraction operator, and then the difference is calculated between the output and the label edge. In this paper, Laplacian operator is used to extract edge features. The formula of edge-aware loss is as follows:

(12) $$\begin{array}{c} L_{SR}^{Edg\;e}=E_{I^{SR}}{\left\|\gamma_{i}\left(G\left(I^{LR}\right)\right)-\gamma_{i}\left(I^{HR}\right)\right\|}_{1}\text{,} \end{array}$$

where *γ*_*i*_(·) denotes an edge extraction method based on Laplacian operator.

#### 3.3.4. Our Composite Loss

Our loss function uses *L*1 loss as the basic loss function, adds perceptual loss to avoid the loss of high-level features, and adds edge perceptual loss to further monitor the integrity of image edge information. The formula is as follows:

(13) $$\begin{array}{c} L_{SR}=L_{SR}^{L1}+\alpha L_{SR}^{Per}+\beta L_{SR}^{Edge}\text{,} \end{array}$$

where *α* and *β* are hyper-parameters.

We use our composite loss to optimize the proposed model, and the algorithm for training the model is shown in Algorithm 1.

## 4. Experiments

### 4.1. Dataset

The IXISR dataset was constructed by Zhao et al. through further processing of IXI dataset [41], which contains three types of MR images: 81 *T*1 volumes, 578 *T*2 volumes, and 578 PD volumes. In this work, we take the intersection of these three types of MR images to obtain 576 3D volumes of each type of MR image. These 3D volumes are then trimmed to 240 × 240 × 96 (*H* × *W* × *D*) to fit the three scaling factors. For SISR, each 3D MR voxel is divided into 96 (*H* × *W*) gray-scale images. LR images are generated based on bicubic downsampling and *K*-space truncation. As for truncation degradation, HR images are first converted to k-space by discrete Fourier transform (DFT) and then truncated along the height and width directions.

### 4.2. Implementation Details

Our method is implemented by using the paddle framework. Similar to the previous work, in the IXISR [41] dataset, we use 70% of the images as the training dataset, 10% as the validation dataset, and 20% as the test dataset. The size of the small batch is set to 16, and the parameter *α* in the loss function is set to 0.3, the parameter *β* is set to 0.1, and the parameter *n* is set to 2. We use a size of 24 × 24 randomly extracted from LR slices and the corresponding HR area. Data enhancement is simply achieved by random horizontal flipping and 90 degree rotation [25]. And millions of iterative trainings are conducted on the NVIDIA GeForce GTX 3090 GPU. We use Xavier initialization [47] and Adam optimizer for all model parameters and an initial learning rate of 0.001 for iterative optimization. Through the optimization of Algorithm 1, a single iteration of the proposed model including all modules takes about one minute. The space complexity depends on the number of parameters involved in the calculation. Specifically, the representation of the number of parameters is reflected in Table 1.

### 4.3. Evaluation Metrics

For quantitative comparison, highly reliable metrics are introduced, such as root mean square error (RMSE), peak signal-to-noise ratio (PSNR), and structural similarity index (SSIM). The calculated metric scores are derived from the comparison of the results *I*_*SR*_ obtained by the super-resolution method and the high-resolution image *I*_*HR*_.

#### 4.3.1. Root Mean Square Error (RMSE)

(14) $$\begin{array}{c} MSE=\frac{1}{HW}\overset{H-1}{\underset{h=0}{\sum }}\overset{M-1}{\underset{w=0}{\sum }}{\left\|I_{HR}\left(h,w\right)-I_{SR}\left(h,w\right)\right\|}^{2}\text{,}\\ RMSE=\sqrt{MSE}\text{,} \end{array}$$

where *h* ∈ [0, *H* − 1] and *w* ∈ [0, *W* − 1] together represent the position of the pixel in *I*_*HR*_ and *I*_*SR*_.

#### 4.3.2. Peak Signal-to-Noise Ratio (PSNR)

(15) $$\begin{array}{c} PSNR=10\times \log_{10}\left(\frac{{\left(2^{n}-1\right)}^{2}}{MSE}\right)\text{,} \end{array}$$

where *n* is the number of bits per pixel value, which generally takes 8.

#### 4.3.3. Structural Similarity Index (SSIM)

(16) $$\begin{array}{c} SSIM=\frac{\left(2\mu_{HR}\mu_{SR}+c_{1}\right)\left(2\sigma_{\left(HR,SR\right)}+c_{2}\right)}{\left(\mu_{HR}^{2}+\mu_{SR}^{2}+c_{1}\right)\left(\sigma_{HR}^{2}+\sigma_{SR}^{2}+c_{2}\right)}\text{,} \end{array}$$

where *I*_*SR*_ is obtained by the super-resolution method and *I*_*HR*_ is the high-resolution image, respectively; *μ*_*HR*_ and *μ*_*SR*_ are the average; *σ*_*HR*_ and *σ*_*SR*_ are the standard deviation; *σ*_(*HR*, *SR*)_ is the covariance of *HR* and *SR*; and *c*_1_ and *c*_2_ are small constants.

### 4.4. Experimental Results

In this paper, the expressiveness of different models is compared in the case of the IXISR dataset (PD, *T*1, and *T*2) of ×2 super-resolution. PSNR, SSIM, and RMSE are used to evaluate the expressiveness of the model. Subdatasets are used under two different sampling (bicubic degradation and truncation degradation) in the dataset. Bicubic downsampling is widely used by LR image generation simulation in SR images, where bicubic downsampling is used to downsample HR images and generate LR images. Truncation degradation is a process that simulates the real image acquisition process. The LR image is obtained by *k*-space truncation, which means that the HR image is intercepted in frequency space for sampling.

Tables 1 and 2, respectively, show the evaluation results of different models of PD, *T*1, and *T*2 datasets under the bicubic downsampling and truncation degradation methods. From Figures 4 and 5, we can see that our model has higher expression ability than other models. Compared with the two residual-based networks SRResNet and EDSR, our module adds PCFB, which helps to improve the performance of the model.

### 4.5. Ablation Studies

The proposed method is based on the improvement of SSResNet, so the ablation experiment will also be carried out around SSResNet. In Tables 3 and 4, we compare the number of parameters and the performance in PSNR, SSIM, and RMSE for all methods. Note that all results are the average values of PSNR, SSIM, and RMSE calculated from MR images on the same dataset. The experimental results show that the proposed method improves the PSNR, SSIM, and RMSE of LR images obtained from BD and TD by 0.2dB, 0.33dB, 0.06dB and 0.17dB, 0.15dB, 0.25dB, respectively, compared with SRResnet, although the amount of parameters is only 0.01MB lower. This shows that PCFB is more effective.

In order to evaluate the effectiveness of the composite loss we constructed, we performed ablation experiments with different loss functions on the PD data in the dataset, as shown in Table 5. Compared with *L*1 and *L*2 loss functions, the PSNR performance of our composite loss function is 0.62dB and 0.56dB higher than that of only using *L*1 and *L*2 loss, respectively, which is a very significant increase. However, there is no significant decrease in RMSE, which only decreases by 0.0013 and 0.0014. In conclusion, the above results show that the loss function designed by us can retain more effective features and provide more reference value for medical applications.

### 4.6. Model Visualization

In order to understand the ability of the proposed model, the model trained in the comparative experiment is used to visually predict the test data. Our method is compared with Bicubic, ESPCNN, VRCNN, SRResNet, and EDSR on the datasets obtained by the two down sampling methods. The visual results are shown in Figures 4 and 5. It can be seen from the enlarged detail feature map that the image reconstructed by Bicubic, ESPCNN, VRCNN, SRResNet, and EDSR methods still has fuzzy distortion to varying degrees, and the visual perception effect is inferior to our method.

## 5. Conclusion and Future Work

High-resolution MR images have smaller voxel sizes, providing clinical physicians with more accurate structural and textural details. However, generating high-resolution MR images usually incurs enormous costs. Image super-resolution is an effective and cost-efficient alternative technique for high-resolution restoration of low-resolution images. In this work, we propose a novel end-to-end MR image super-resolution method. First, we introduced a parameter-free block fusion block (PCFB) that can split the feature map into *n* branches for better fusion features without parameters. Second, a training strategy combining perceptual loss, gradient loss, and LI played an important role in accelerating model fitting and improving prediction accuracy. Finally, the proposed method is effective in the super-resolution task of MR images, improving model accuracy. Our future work needs to focus more on lightweight processing of the model to reduce the model's parameters while achieving the optimal model accuracy mentioned in the paper.

## Figures and Tables

**Figure 1:** The proposed architecture of super-resolution. The architecture mainly includes the parameter-free chunking fusion block (PCFB) model, residual block, and reconstruction block. The residual block consists of convolutions, activation functions, and skip connections. PCFB divides the feature map into *n* branches through a split channel, and each branch is fused after passing SimAM to obtain parameter-free attention feature enhancement. The reconstruction block consists of 3 × 3 convolution, 1 × 1 convolution, PReLU, and the PixelShuffle layer.

**Figure 2:** Parameter-free attention module.

**Figure 3:** PixelShuffle.

**Figure 4:** Super-resolution reconstructed LR images are obtained by bicubic downsampling (BD). The figure shows the visual comparison of other methods with our proposed method.

**Figure 5:** Super-resolution reconstructed LR images are obtained by *k*-space truncation (TD). The figure shows the visual comparison of other methods with our proposed method.

**Algorithm 1:** Training framework based on the proposed method.

**Table 1:** The super-resolution reconstructed LR image is obtained by bicubic downsampling (BD). The experimental data show the comparison of other methods with our proposed method in various evaluation indexes: PSNR, SSIM, and RMSE.

	Bicubic downsampling (BD)									
	PD			*T*1			*T*2			Params (MB)↓
	PSNR↑	SSIM↑	RMSE↓	PSNR↑	SSIM↑	RMSE↓	PSNR↑	SSIM↑	RMSE↓	—
Bicubic	32.63	0.9675	0.0243	32.10	0.9542	0.0256	32.71	0.9601	0.0236	—
ESPCNN [42]	32.07	0.9647	0.0259	31.52	0.9514	0.0271	32.03	0.9555	0.0253	0.22
VRCNN [48]	33.67	0.9743	0.0217	32.84	0.9632	0.0236	34.37	0.9713	0.0196	**0.21**
EDSR [25]	34.40	0.9782	0.0204	33.03	0.9651	0.0231	35.51	0.9756	0.0173	5.08
PAN [49]	34.33	0.9783	0.0203	33.10	0.9652	0.0230	35.37	0.9759	0.0176	0.72
NAFNet [50]	32.53	0.9676	0.0248	31.97	0.9551	0.0263	32.63	0.9594	0.0239	16.58
Proposed	**34.52**	**0.9790**	**0.0199**	**33.23**	**0.9659**	**0.0227**	**35.53**	**0.9761**	**0.0173**	5.27

Bold values highlight the optimal results.

**Table 2:** The super-resolution reconstructed LR image is obtained by *k*-space truncation (TD). The experimental data show the comparison of other methods with our proposed method in various evaluation indexes: PSNR, SSIM, and RMSE.

	*k*-space truncation (TD)								
	PD			*T*1			*T*2		
	PSNR↑	SSIM↑	RMSE↓	PSNR↑	SSIM↑	RMSE↓	PSNR↑	SSIM↑	RMSE↓
Bicubic	32.34	0.9555	0.0252	31.65	0.9361	0.0270	32.36	0.9477	0.0246
ESPCNN [42]	31.73	0.9525	0.0270	31.02	0.9273	0.0287	31.71	0.9427	0.0263
VRCNN [48]	32.86	0.9621	0.0238	32.10	0.9452	0.0257	33.67	0.9613	0.0213
EDSR [25]	34.14	0.9736	0.0209	32.70	0.9529	0.0240	35.49	0.9724	0.0174
PAN [49]	33.86	0.9726	0.0216	32.75	0.9580	0.0240	35.05	0.9703	0.0183
NAFNet [50]	32.32	0.9574	0.0252	31.67	0.9395	0.0269	32.42	0.9523	0.0244
Proposed	**34.20**	**0.9752**	**0.0208**	**32.87**	**0.9591**	**0.0238**	**35.66**	**0.9734**	**0.0172**

Bold values highlight the optimal results.

**Table 3:** Performance and parameter comparison of the proposed module. The super-resolution reconstructed LR image is obtained by BD.

	Residual block	Reconstruction block	PCFB		PSNR↑	SSIM↑	RMSE↓	Params (MB)↓
SRResnet [51]	✓	✓	—	PD	34.32	0.9783	0.0203	5.28
				*T*1	32.90	0.9636	0.0234	
				*T*2	35.47	0.9761	0.0174	

Proposed	✓	✓	✓	PD	**34.52**	**0.9790**	**0.0200**	**5.27**
				*T*1	**33.23**	**0.9659**	**0.0227**	
				*T*2	**35.53**	**0.9761**	**0.0173**	

Bold values highlight the optimal results.

**Table 4:** Performance and parameter comparison of the proposed module. The super-resolution reconstructed LR image is obtained by TD.

	Residual block	Reconstruction block	PCFB		PSNR↑	SSIM↑	RMSE↓
SRResnet [51]	✓	✓	—	PD	33.97	0.9718	0.0212
				*T*1	32.72	0.9525	0.0241
				*T*2	35.41	0.9726	0.0177

Proposed	✓	✓	✓	PD	**34.14**	**0.9752**	**0.0209**
				*T*1	**32.87**	**0.9591**	**0.0238**
				*T*2	**35.66**	**0.9734**	**0.0172**

Bold values highlight the optimal results.

**Table 5:** Comparative experimental results of the introduced loss function.

	*L*1 loss	*L*2 loss	Composite loss	PSNR↑	SSIM↑	RMSE↓
Ours	✓	—	—	33.89	0.9763	0.0214
Ours	—	✓	—	33.96	0.9772	0.0213
Ours	—	—	✓	**34.52**	**0.9790**	**0.0200**

Bold values highlight the optimal results.

## Data Availability

The IXISR dataset used to support the findings of this study are included within the article [41].
